The article "Evaluation of the Effect of Intensive Nursing Intervention Based on Process Analysis" was retracted in 2022. Reason: concerns about the peer review.

# Evaluation of the Effect of Intensive Nursing Intervention Based on Process Analysis

**DOI:** 10.1155/2021/8769780

**Published:** 2021-12-06

**Authors:** Zhiying Zhang, Huiju Zhu

**Affiliations:** Department of Critical Medicine, The First Affiliated Hospital of Soochow University, Suzhou City, Jiangsu Province 215000, China

## Abstract

In order to achieve significant improvements in the evaluation of key indicators such as speed, quality, cost, and service, this paper fundamentally rethinks and completely redesigns the business process, and recreates a new business process. This study combines the particularity of AMI with emergency nursing to construct an in-hospital AMI emergency nursing process to further standardize the AMI rescue work. The implementation of the process helps to clarify the responsibilities and requirements of nurses in the AMI emergency process, reduce the delay time of AMI emergency, and improve the efficiency and effectiveness of emergency. In addition, after refactoring the business process, this paper builds an intelligent digital critical illness monitoring system. This system combines the original work flow of the ICU medical staff, optimizes the work flow of the medical staff through computer technology and information technology, and designs and completes the digital intensive nursing system software to run and use in the hospital and obtain significant results.

## 1. Introduction

Nursing quality is an important indicator to measure the quality of nursing staff, the level of nursing leadership management, nursing business skills, and work results, and it directly reflects the professional characteristics and work connotation of nursing work. Since the reform and opening up, nurses have continuously improved their own quality, explored the best service model, and made many efforts to improve service quality. However, the satisfaction survey of nursing quality is not ideal, and many disputes are complaints about nursing [1]. In recent years, the specialized technology of intensive nursing medicine has been continuously developed, but in the absence of a unified ICU nursing quality evaluation standard in China, the quality of ICU nursing has stagnated, which has greatly affected the quality of hospitals.

During the last decade, there have been many shifts in how we think about ICU nursing quality. When used to gauge the quality of ICU care, certain indicators, including as cure rates, death rates, length of stay, and the usage of specific equipment indicators (such as the pulmonary arterial catheter), have flaws and limits that make them unreliable. As a result, new ideas for evaluating nursing quality have emerged in recent years, the most well known of which being Berick's “4 objectives” theory of nursing quality. He said that evaluating the quality of medical nursing care in any context should include the following four goals [2]: (1) impact assessment of nursing practice is the bedrock and cornerstone of medical nursing; it is necessary to evaluate the nursing effect of all patients as well as individual differences, so as to better reflect the effect of nursing practice; (2) the appropriateness of nursing work, that is, “what kind of nursing work to carry out,” which includes professional nursing guidance and the formulation of reliable nursing operating procedures; (3) the implementation of nursing measures, that is, “how to do a good job in nursing,” means to fully mobilize all aspects of nursing and give full play to the potential of each nursing unit; (4) the purpose of nursing is to explain the “value of nursing,” which is evaluated by individuals and the public as a whole. Among the above 4 goals, the implementation of nursing measures is one of the most commonly used indicators for hospitals to improve the quality of ICU nursing.

My nation has made some strides in nursing theory research in the last several years. There is growing interest among nursing managers in incorporating contemporary management theories into their day-to-day work, and they are exploring new ways to do so within the context of conventional empirical management in their nation. This is a significant advancement in the development and enhancement of nurse quality management in the United States. As quality awareness has increased, many hospital nursing managers have gradually integrated system theory and behavioral science concepts and procedures into nurse quality management.

## 2. Related Work

The construction of sensitive indicator systems for ICU nursing quality abroad is relatively mature. Some countries or regions have formed national-level ICU nursing quality evaluation indicators, such as the United States, the Netherlands, Germany, India, Taiwan, the United Kingdom, and Spain. Moreover, many studies on nursing quality indicators start from “why should ICU nursing quality indicators be established.” In the end, most researchers [3] regard nursing should be safe, effective, timely, patient-centered, efficient, and fair as the framework for developing nursing quality indicators. The literature [4] built an index system that can measure the quality of nursing in all areas of the ICU based on the “structure-process-outcome” theory. Research [5] utilised process indicators to create an index of intensive care unit (ICU) quality. Analyzing data has shown a reduction in ICU hospitalisation length, morbidity, and death for patients getting standardised monitoring process indicators. For the European Association for Intensive Medicine, nine quality indicators for intensive nursing were developed by an expert committee consisting of 18 specialists from nine countries. There are three structural indicators included in this report: ICU bed-to-nursing ratio, 24-hour availability of ICU doctors, and 2 process indicators related to the adverse event reporting system and 4 outcome indicators, namely, standardized mortality rate, ICU 48-hour return rate, central venous catheter-related bloodstream infection rate, and unplanned extubating rate [6]. The literature [7] formulated 139 indicator systems according to the actual development of the hospital and divided them into outpatient, emergency, inpatient, and ICU nursing quality modules. The ICU nursing quality indicators constructed in the literature [8] are the most common, emphasizing morbidity, mortality, and patient safety, but their operability, specificity, scientificity, and sensitivity require further evaluation. Because different countries and regions have different understandings of the definition of the nursing quality sensitivity index and its connotation, it leads to the choice of various indexes with different tendencies.

Literature [9] follows the TQM concept and applies the PDCA cycle to continuous nursing quality management. After implementation, nursing quality and patient satisfaction have been improved. The literature [10] demonstrates how to utilize the “Z-type management theory” to direct nursing work and enhance overall nursing job quality and how to apply the “flexibility principle” to quality assessment criteria, utilize the “human-centered concept” to help managers develop a more holistic management style, and utilize the “expectation theory” to elicit the passion and inventiveness of nursing staff and to encourage nursing quality improvement. By utilizing the “dynamics” principle, nursing management functions are strengthened, ensuring that nursing management is always in a state of continuous development and relative stability; by utilizing the “closed principle,” nursing management functions are strengthened, ensuring that nursing management operates normally and effectively inertially. With the improvement of national laws and regulations, people's self-protection and legal awareness have been continuously enhanced, and “crisis management” has been applied to nursing management in recent years. “Crisis management” enhances nurses' crisis awareness and improves nurses' service awareness and the quality of nursing work [11]. Hospital managers are now focused on “risk management.” When used in conjunction with ICU nursing quality management, nursing risk management almost ensures the highest level of nursing care. To improve nursing quality, “incentive theory” may mobilise nurses' subjective initiative as a foundation for nursing management [12]. Nursing quality management has now reached a new level, thanks to all of these contemporary management ideas. Experience-based quality control is no longer the foundation.

Literature [13] incorporated nursing expenditure-related indicators into the indicator system and established an ICU nursing quality evaluation indicator system covering three aspects: element quality, link quality, and terminal quality. Literature [14] established 3 first-level indicators, 12 second-level indicators, and 74 third-level indicators from three aspects: basic evaluation, process evaluation, and result evaluation based on the current status of the core competence of ICU nurses. Literature [15] established 3 first-level indicators, 22 second-level indicators, and 77 third-level indicators, which emphasized the scientific view of terminal quality. Literature [16] developed 28 distinct assessment indicators from six aspects: basic nursing quality, nursing safety quality, nursing management quality, disinfection and isolation quality, nursing document quality, and end-of-life nursing quality. Literature [17] from the perspective of nursing safety combined with local hospital conditions used the “structure-process-outcome” model to establish 3 first-level indicators, 21 second-level indicators, and 97 third-level indicators. The indicator system is mainly used for evaluation, safety, and quality of ICU care. Literature [18] established a total of 32 evaluation standards for safety and quality of care in intensive care units with two levels. Literature [19] produced data-driven ICU nursing quality management indicators that were based on the real condition of the hospital and the viewpoint of nursing management. Literature [20] developed 20 parameters of ICU nursing quality based on evidence-based theory. Literature [21] establishes a framework for evaluating the quality of ICU nursing care based on the principle of exceptional performance.

## 3. Method

According to the guidance of the BPR theory S-A framework diagram (as shown in Figure 1), the working procedures of design reengineering are as follows: (1) initiation: in this step, a process reengineering team is formed, principles are clarified, and goals are drawn up; (2) preliminary construction: a. modeling of original working procedures; b. analysis, diagnosis and redesign; (3) continuous improvement: this step is pretested, and Delphi expert consultation is conducted to continuously improve the process; (4) process evaluation: in this step, the actual application effect of the process after reengineering is evaluated.

According to the requirements of the BPR theory, the reengineering team should be composed of a leader as the core and 5-20 other experts in related fields as the assistance. In this study, the members of the process reengineering team included the vice president of the hospital, the director of the nursing department, the head nurse of the emergency department, the head nurse of the cardiology department, the head of the chest pain center, emergency doctors, emergency nurses, and other relevant personnel. The vice president of the hospital, in his or her capacity as reengineering organiser, is in charge of overseeing the whole research process from start to finish. The director of the nursing department and the emergency room and cardiology department's head nurses all have extensive managerial and clinical backgrounds. They constitute the backbone of the reengineering process and may offer significant support for process analysis and rearrangement. Having the chest pain center's manager acquainted with center's operations as well as its assessment indicators is critical to study's success. The construction of the critical emergency nursing process based on the chest pain center further enhances its spread ability. The critical and emergency medicine knowledge and clinical experience of emergency doctors have enhanced the professionalism and pertinence of this process. Emergency nurses are the direct users of this process, and their clinical experience and insights are the guarantee of the operability of this process. We determine the principles of process reengineering: (1) patient-centered; (2) safety-based; (3) fast and efficient process operation as the goal; (4) continuous improvement as the concept. The goals of process reengineering were formulated: (1) after reengineering, the process has strong operability, which can ensure the smooth progress of the intervention of critically ill emergency nursing, the efficiency of rescue work is high, and the delay time of emergency for critically ill patients is reduced. (2) The scope of work for nurses in the critically sick emergency process is defined via process reengineering, and medical nursing and nursing coordination is enhanced through this approach. A defined time and responsibility structure is developed after rebuilding to lessen the reliance of critical emergency nursing on experienced emergency nursing staff (3). (4) The reengineered process needs to run on the basis of the original process and be stable and smooth and does not conflict with the existing overall system or other single department systems.

At the moment, there is no foundation for critical emergency nursing process standards, and nurses in different institutions do critical emergency nursing based on their own experience, with comparable job content. A hospital in Hangzhou is a class A general hospital with the most comprehensive level of care among Zhejiang Province's hospitals. In 2017, the hospital completed the accreditation process for chest pain centers and was given the chest pain center demonstration unit. It provides an excellent platform for urgent emergency situations. Therefore, this paper takes the hospital as an example and combines literature analysis, previous case analysis, and field investigations to use business flowcharts to simplify and model its critical emergency nursing work (Figure 2).

It is split into three parts: triage, emergency, and transfer for analysis. Several important nodes are acquired. Preexamination, communication, and preparation are all important nodes in the triage process. In an emergency, the most important things to focus on are survival, diagnosis, treatment, and communication. Patient preparation, equipment and supplies, communication, and handover of the condition are all critical nodes in the transfer process. This is followed by layer-by-layer refinement of each critical node to uncover process's most minute details. Finally, 11 key nodes and 29 detailed nodes are extracted (as shown in Figures 3, 4, and 5). After that, we perform one-by-one analysis to find out the problem and give a corresponding solution strategy.

Individual complicated issues are replaced into the fishbone diagram based on the findings of the node analysis to assist further investigation of problems' likely causes. A draft procedure is created based on the findings of the fishbone diagram analysis to aid in clarifying the objective and substance of the interview during a semistructured interview. As seen in Figures 6, 7, and 8, this article uses lengthy triage times, inaccuracies in triage, and repetitive tasks as examples.

We conduct relevant training and assessments for nurses to ensure the effective implementation of the process and test its true effects. The training content is as follows: (1) ECG training: nurses need to be familiar with how to use all models of ECG machines in the hospital and the meaning of relevant signs. Nurses need to master the detection position of the 12 and 18 lead ECG. Nurses need to master the identification of basic electrocardiograms, such as STEMI, NSTEMI, ventricular fibrillation, atrial fibrillation, and normal electrocardiogram, and understand the corresponding infarct position on the electrocardiogram. Nurses need to master the possible interference factors and coping methods in the application of electrocardiograph. (2) Nurses must comprehend the primary content of critically ill patients' condition observation, understand the rationale for critically ill patient triage, and understand the procedure for assessing the risk of critically sick patients. The training will take the form of short seminars, with the instructors being the director of hospital's ECG room and cardiologists. Assessment form: (1) the ECG training will be assessed in the form of a combination of operation and volume. (2) The condition observation is assessed in the form of a combination of roll-out and ward rounds. Every nurse in the emergency department must pass an assessment.

The essential time nodes of each patient are recorded using an electronic automated timing system. Time management and electronic automated timing are used in the data input process. If anything goes wrong, we will fall back on the electronic automated timing system. We utilise two-person input and verification to convert the time data into a value in minutes. A nonparametric test was used to examine differences between groups that were not normally distributed, whereas a *t* test was used to compare those differences that were not normally distributed.

## 4. Intelligent Digital Critical Nursing Monitoring System

On the basis of the above analysis, we build a digital monitoring system for critical nursing. The purpose of system development is to use computer technology, database technology, and software engineering approaches to create high-performance, highly integrated, and highly available digital intensive nursing information system computer software for the intensive care unit. Simultaneously, it undertakes extensive research on how to implement automated extraction of medical orders and the template for nursing medical records, data exchange, and ICU digital administration. The digital intensive nursing system comprehensively manages the various clinical work links of ICU medical staff, standardizes and automates ICU work, and reduces the time for ICU nurses to record patient signs and manually operate medical documents and nursing records, improve work efficiency, and realize digital management of ICU.

Medical advice processing, nursing papers, pipeline/incoming and outgoing records, and query statistics are all part of the digital intensive care system. When it comes to medical orders, we have to deal with both long-term and short-term orders. When it comes to nursing papers, we use a critical scoring system, template writing, and automated production. Data Query Statistics Module: Ward Skin Test Medical Order Queries, Long-Term Drug Execution Form Printing Summary by Execution Method Printing Medical Order Form Queries, etc. Basic features like user administration and dictionary data maintenance are also included in the system

In the information age, information and data security is regarded as one of the core issues in software development. As an important part of the hospital, ICU needs to deal with a large amount of data and information every day. How to deal with data security issues is required in the software development process. Consider it all. During the process of data transmission, there are risks of loss, omission, tampering, etc. To avoid these circumstances and to protect the security of data and information, the system should assign relevant permissions to distinct roles and functional modules to limit access. It conducts business within the boundaries of the appointing authority. Each user attempting to access the system must be authenticated. Different system roles have access to just a subset of function modules. Under the distribution of system permissions, the corresponding interface functions can be used after verification.

Every day, the hospital deals with a significant quantity of patient data, and the intensive care unit is no exception. Engineering a computerised intensive nursing system from scratch is no small feat. You will need to be familiar with computer science, database design, and information systems. So, the digital intensive nursing system must be adjusted based on these real-world circumstances in order to cope with the processing of huge quantities of data. The equivalent top-level data flow diagram, illustrated in Figure 9, may be produced based on system need and business process analysis.

This system uses a mixed architecture of C/S and B/S. In the C/S (Client/Server) system architecture, Client and Server are often located on two computers with farther physical space. First, the Client program submits user's request to the Server program, and the Server program receives the request from the Client program. After that, the corresponding processing is made, and the processing result is returned to the Client program. Finally, the Client program presents the returned result to the user in a certain way. The C/S architecture has strong transaction processing and data manipulation capabilities, simple structure, and easy to be accepted by people. However, with the continuous improvement of software complexity, the disadvantages of C/S architecture, such as high system development cost and difficulty in software maintenance and upgrading, have gradually been exposed. B/S (Browser/Server) architecture, that is, browser and server architecture, is a change or improved structure of the C/S architecture with the rise of Internet technology. Under this architecture, the user interface is implemented through a browser, a small part of the work is performed on the front end (Browser), and the main transaction logic is implemented on the server side. This greatly reduces the burden on the client computer, reduces the cost of system maintenance and upgrades, and reduces the overall cost of users. However, compared with the C/S system architecture, the B/S system architecture also has many shortcomings. For example, the B/S architecture lacks the ability to support dynamic pages and does not integrate effective database processing functions. Therefore, the software system using the B/S architecture is far inferior to the software system of the C/S architecture in terms of the response speed of data query and statistics. Moreover, the software system of the B/S architecture has poor scalability, and security is not easy to control. This system combines the two system architectures of B/s and C/S to maximize their strengths and avoid weaknesses, effectively exerting their respective advantages. The medical order processing module has higher requirements for data processing and response speed, so the medical order processing module of this system adopts the C/S architecture. The back-end processing of functions such as patient nursing medical records, pipelines, and access records is complicated. In order to avoid the bloat of the client, these functional modules adopt the B/S architecture system.

These devices are all connected by way of a wireless router and mobile terminal via system's network. In addition, this hospital's ICU ward's beds are equipped with four network connections and use a central collecting mode. A central monitoring system host collects data from the switch, which is linked to the equipment through a local area network. There is also an intensive nursing workstation built into every ICU bed, and a high-speed wireless router on top of the ICU ward provides coverage for the whole ICU ward's wireless network. According to Figure 10, the mobile device at patient's bedside may connect to the server via a wireless network.

After constructing the above system, the method and system proposed in this paper are evaluated for the effect of intensive nursing intervention, and the system effect is evaluated by the survey interview method, and the results shown in Table 1 and Figure 11 are obtained.

The above research shows that the critical nursing intervention method and digital monitoring system based on process analysis proposed in this paper have good results.

## 5. Conclusion

This study uses the BPR theory to construct the in-hospital critical emergency nursing process, effectively reduces the delay time of first aid for critically ill patients, improves the emergency response effect of patients, and improves the efficiency of emergency nurses' rescue work, which helps to solve the current dilemma faced by intensive nursing work. By combining the traditional ICU staff work flow with computer technology and information technology, this method maximizes medical personnel's efficiency. Furthermore, the software for the digital intensive nursing system developed and finished in this article has shown amazing results in operation and use in hospitals. Medical personnel in the critical care unit use a computerised intensive nursing system to keep track of their different clinical tasks. Moreover, it realizes functions such as automatic transfer of medical advice and intelligent reminders, electronic writing of nursing documents, records, and statistics of pipelines and in-outs, and data sharing with HIS, LIS, and PACS. In addition, it reduces the repeated transfer of data and manual operations, reduces the workload of the ICU medical staff, improves work efficiency, and realizes the digital management of the ICU.

## Figures and Tables

**Figure 1:** Process reengineering S-A framework diagram.

**Figure 2:** The original flow chart after modeling.

**Figure 3:** Triage node.

**Figure 4:** Emergency node.

**Figure 5:** Transfer node.

**Figure 6:** Fishbone figure 1: long triage time.

**Figure 7:** Fishbone figure 2: inaccurate triage.

**Figure 8:** Fishbone figure 3: repetitive work.

**Figure 9:** Top-level data flow diagram of the digital intensive nursing system.

**Figure 10:** System network architecture.

**Figure 11:** Statistical diagram of intensive nursing intervention data based on process analysis.

**Table 1:** Evaluation of the effectiveness of intensive nursing intervention based on process analysis.

Number	Evaluation	Number	Evaluation	Number	Evaluation
1	90.07	22	92.54	43	92.19
2	86.40	23	90.24	44	87.05
3	90.62	24	90.10	45	92.78
4	90.65	25	92.68	46	89.43
5	92.54	26	86.41	47	91.34
6	91.36	27	89.16	48	93.38
7	96.53	28	93.03	49	91.33
8	91.89	29	94.28	50	86.66
9	94.90	30	91.28	51	89.86
10	91.47	31	91.74	52	92.56
11	95.40	32	88.46	53	91.69
12	92.58	33	88.77	54	92.83
13	90.92	34	91.75	55	96.49
14	94.54	35	95.27	56	94.04
15	91.89	36	90.27	57	91.54
16	89.09	37	88.24	58	92.23
17	96.57	38	93.33	59	92.70
18	95.06	39	89.43	60	90.40
19	88.68	40	86.98	61	96.00
20	96.99	41	91.63	62	92.47
21	88.56	42	90.20		

## Data Availability

The data used to support the findings of this study are included within the article.
